This article has been retracted.

# Innovative Practice of Multimusic Performance Culture Education of Core Literacy in Multimedia Environment

**DOI:** 10.1155/2022/9440849

**Published:** 2022-07-30

**Authors:** Siyuan He, Sixian He, Xin Gao

**Affiliations:** ^1^College of Music, Ningxia University NXU, Yinchuan 750021, Ningxia, China; ^2^Faculty of Music and Performing Arts, Universiti Pendidikan Sultan Idris UPSI, Tanjong Malim 35900, Perak, Malaysia; ^3^College of Music and Dance, North Minzu University NMU, Yinchuan 750021, Ningxia, China; ^4^School of Materials Science & Engineering, North Minzu University NMU, Yinchuan 750021, Ningxia, China

## Abstract

Under the framework of disciplinary knowledge integrating technology, the multimedia teaching application of music performance attracts a major opportunity for reflection and reconstruction. The purpose of this study is to explore the laws and experiences of music performance teachers' multimedia teaching applications under the framework of subject teaching knowledge integrating technology. Through the research to understand the classroom multimedia teaching application of music performance teachers, according to the research results, relevant strategies are put forward for the application of music performance teachers' classroom multimedia teaching, in order to effectively improve the classroom teaching effect of music performance teachers. This research mainly uses the classroom observation method and data statistical analysis method and takes 100 music video lessons of the National Educational Resources Public Service Platform as the survey object. A total of 100 teachers were observed and scored in the classroom through the compiled multimedia teaching observation table for music performance teachers, and then the data was analyzed to draw conclusions. The conclusions of this study are as follows: The multimedia application behaviors of the teachers of the excellent courses are different from those of the teachers of the daily classes. The two types of teachers have differences in the effectiveness of multimedia teaching application of music performance, and the scores of the practical application of information technology are uneven. The overall score of multimedia teaching applications of excellent course teachers is higher than that of daily course teachers, and the classroom teaching effect is better. In this regard, based on the observation and assessment of the effectiveness of multimedia teaching applications by two types of teachers, this paper puts forward some suggestions for music performance teachers to improve the effectiveness of multimedia teaching applications in classrooms from the aspect of teachers themselves and educational functions. It is hoped that it can provide some theoretical basis and practical materials for the personal and professional development of music performance teachers.

## 1. Introduction

Multimedia technology is an important part of modern information technology. Its characteristics and achievable functions are very suitable for the needs of music performance teaching. Using multimedia, teachers can integrate beautiful songs, dynamic pictures, and rich emotions. In the influence of the music situation created by the teacher, the charm conveyed by the music can be more intuitively felt, which has a positive effect on improving the aesthetic ability of college students [1]. From this advantage, the teaching design based on multimedia technology should combine the cognitive laws of college students, the different characteristics of multimedia technology, and the subject characteristics of music performance to improve and optimize the teaching content, to enhance the interest of college students in learning music, and inspire college students to learn more about music. Creative thinking, deepening students' perception of music, and understanding music emotions put students in the situation, in order to cultivate their aesthetic ability. Therefore, this paper attempts to introduce multimedia technology into the teaching of music performance courses, using interview methods, field investigation methods, etc., to first understand the current status of music performance teaching, and on this basis, enrich teaching methods, improve teaching efficiency, and pay attention to students' individualization [2].

College music performance education is an important way to implement aesthetic education, and it is also one of the ways to cultivate college students' humanistic quality. Music can cultivate people's sentiments, and the culture behind the music can enrich their minds, help students establish correct their views, and cultivate eyes to discover beauty. The way of thinking and habits need to be cultivated from an early age. The university stage is in the period of students' concept formation, so university music performance education plays a decisive role [3]. For the artistic pursuit of college students, high-quality music teaching can play a huge role in promoting college students to have a higher appreciation ability, and at the same time, it can make them have higher requirements for themselves, and promote their aesthetic ability not only for judging things but also is also an important measure to measure one's progress [4]. With aesthetic ability, students have critical expression ability, which can encourage introverted and extroverted college students to express their inner feelings and judgments about music bravely, and promote their ability to communicate in the future society [5].

In 2005, based on the importance of subject teaching knowledge, considering the wide application of information technology in classroom teaching, and on the basis of valuing teaching content knowledge (PCK), L. Yan [6] first put forward the view that technology, teaching method, and subject content should be combined. (Technological Pedagogical Content Knowledge, referred to as TPCK). To facilitate memory and highlight the overall meaning of teachers' knowledge, TPCK was later renamed TPACK (Technological Pedagogical and Content Knowledge). This new conceptual framework describes in detail the integrated knowledge teachers should have in the information environment and provides information technology and content knowledge for teachers. The development of subject curriculum integration ability provides theoretical guidance [7].

TPACK [8] is the basic knowledge that teachers should have in the information age. Teachers must have a deep understanding of the relationship between information technology, pedagogy, and subject content. It directly affects the ability of teachers to apply information technology. This research will be based on the TPACK knowledge framework and combined with the music discipline to study the application status of multimedia teaching for primary school music teachers. The results can theoretically enrich the TPACK knowledge framework and in practice can promote music teachers to reflect on and improve their knowledge structure. Dadi promotes the research on teacher integration technology and promotes the professional development of teachers.

## 2. State of the Art

### 2.1. Overview of Foreign Research

In 1963, Stanford University in the United States started the research on multimedia technology-assisted teaching and then cooperated with IBM to develop the IBM1500 teaching assistance system, which was the first country to conduct multimedia technology-assisted teaching research. Shen and Renee [9] believed that multimedia technology should be used to assist teaching practice, in other words, he proposed multimedia technology as a tool to assist teaching [10]; Deng believed that multimedia technology was very important in middle school practice. It can be used as a tool to enhance students' interest and fully arouse students' enthusiasm for learning [11]; Fan believes that in the process of multimedia technology-assisted teaching, teaching purposes and methods are issues that need to be carefully considered by teachers [12]. In order to more accurately understand the characteristics and effects of multimedia technology as a high-level cognitive tool, educational psychologists have done a lot of related experiments [13]. Norman studied the characteristics of “construction” and “carrier” of multimedia technology and their relationship with teaching objectives [14]; Guo conducted a comparative study on the presentation effects of text media and animation media [15] and found that the effect of using multimedia technology not only has significant individual differences but also different types and characteristics of media. The joint use can get a better effect. In 1997, Lappe [16] published “Multimedia Learning: Are We Asking the Right Questions,” which stimulated the research enthusiasm of scholars in related fields for multimedia technology-assisted learning. In 2001 and 2005, he published “Multimedia Learning,” respectively, [17] and “Multimedia Learning Handbook,” [18] which mainly explain the prospects, related theories, and cognitive principles of multimedia technology-assisted learning.

Judging from the above research status, multimedia technology-assisted teaching has received early attention abroad, and has been highly valued by scholars. For example, developed countries such as the United States and the United Kingdom also pay more attention to the auxiliary functions of multimedia in teaching practice research. Practical courses are also very representative. In short, all countries in the world are paying great attention to multimedia technology-assisted teaching, including its development, practice, and optimization. Multimedia has also attracted great attention from scholars in the educational field.

### 2.2. Overview of Domestic Research

The sprout of electronic education in my country is that He Kekang proposed that multimedia technology can assist teaching and optimize the teaching mode through this technical means [19]. Electronic education refers to a form of education that uses projection, slide show, audio recording, video recording, radio, film, TV, computer, and other technologies to transmit educational information, and design, study, and manage this process. It is an effective way and method to promote school education and teaching reform and improve the quality of education and teaching. It is an important part of realizing the modernization of education. At the same time, many educational institutions began to use projectors, PPTs, and other media for teaching. After that, more and more domestic scholars began to study multimedia teaching. Huang et al. put forward the application prospect of information technology in middle and university education. In order to maximize the role of multimedia technology in high school education [20], described a biological learning model based on multimedia technology and explained its ideas and implementation methods; Ke Heping (2002) proposed a multimedia teaching resource library and a network learning resource library and constructed several multimedia teaching resource libraries and network learning resource libraries; proposed the auxiliary role of multimedia technology in teaching at an early stage in China. She believes that the application of multimedia technology in teaching dilutes people's subjective consciousness and is too mechanized; in the study of through experimental research according to the analysis multimedia teaching needs to follow the characteristics of students' cognitive development, and the principles of multimedia teaching design need to be constantly tested and improved in teaching practice and adjusted according to the feedback effect of students; The teaching effect presented at the same time as auditory is better, so in multimedia teaching, visual and auditory representations should be used at the same time, not one-sided. The problem of thinking ability cannot stop at the level of knowledge; believes that the application of multimedia technology in music teaching in colleges and universities can add teaching content, expand learning resources, and enrich teaching methods, thereby improving teaching quality; sorts out and compares Meyer's theory and further analyzes its multimedia teaching principles. He thinks that Meyer's theory has a positive effect on students' understanding of knowledge.

To sum up, although the research on multimedia technology-assisted teaching in China started late, the development progress and speed are very fast, and the pertinence is stronger. With the development of information technology, there are more and more research studies on the application of multimedia technology in teaching, but specific research on the multimedia application in music performance courses is not much, nor is it in-depth enough. Therefore, this research applies multimedia technology to music performance courses and constructs a teaching model and teaching design for it.

## 3. Methodology

### 3.1. Research Design and Architecture

Through further thinking on this research question, the basic research structure of this paper is drawn as follows.

This paper adopts the classroom observation method, data statistical analysis method, and other research methods and focuses on the effect of multimedia teaching application on music performance. Different teachers adopt different application modes for multimedia teaching, so their influence on the teaching effect of music performance is also different. Finally, the research conclusions and reflections are made, and some practical teaching suggestions are put forward on relevant research issues as shown in Figure 1.

The preliminary structure is drawn as follows.

### 3.2. Research Methods and Objects

#### 3.2.1. Research Methods

*(1) Classroom Observation Method*. By observing the excellent courses and daily courses of the Music Performance Department, and recording statistical related data in detail, we can analyze the influence of teachers' classroom multimedia teaching application behavior mode on classroom teaching effectiveness.

*(2) Statistical Analysis of Data*. Implement the measurement tool to obtain the relevant data of the multimedia teaching application of music performance teachers and organize the obtained data, and then process and analyze the data with the help of SPSS, Excel, and other software.

#### 3.2.2. Research Objects

The application of TPACK focuses on practical operation and application effects. In the selection of research objects, first of all, it needs to be universal, the number of samples should be large, and the general laws of the data should be reflected through the observation of multiple samples; secondly, there should be differences, and the samples of the class should be selected. There must be a gap in the level; again, it is necessary to have contrast, and it is not realistic to compare the teaching performance of the same classroom. Therefore, this study conducts a comparative analysis from different sample levels of the same teaching content to increase the reliability and accuracy of the data inspection. The specific framework is shown in Figure 2.

The National Educational Resources Public Service Platform (1s1k.eduyun.cn) “one teacher for one excellent course, one teacher for one lesson” activity is jointly organized and implemented by the Second Department of Basic Education of the Ministry of Education and the Central Electronic Education Center. The purpose is to mobilize the majority of middle and university teachers, use the enthusiasm and creativity of information technology to promote the deep integration of multimedia and education and teaching, and improve the quality of education and teaching. The author believes that the lessons included in this platform are cutting-edge and authentic, and to a certain extent ensure their representativeness. Based on the above situation, the research object of this research is finally confirmed as the sample of 50 music department excellent courses and 50 music daily lessons on the website of the National Educational Resources Public Service Platform One Teacher One Excellent Course website (1s1k.eduyun.cn). Analysis and comparison of excellent courses and daily courses in the same section of the version: In order to ensure the quality of course selection, the excellent courses selected for the study are the 2017–2019 excellent courses; the daily course selection is the most viewed course on the website before the author's research node in 2017–2019.

### 3.3. Reliability and Validity Analysis

In order to make the content design of the form as comprehensive as possible, we discussed with the instructor and three teachers with high influence in the field of music education, mainly the rationality of the structure, content sufficiency, and evaluation of the “Classroom Observation Record Form.” Suggestions on the accuracy and effectiveness of the contents of the form should be reviewed for completeness.

Based on the “Classroom Observation Record Form” after expert validity, the researchers first used the Cronbach's alpha coefficient method to analyze the reliability of the scale after observing and evaluating the scores of 100 music performance classes. The result is as shown in Table 1.

The results of the report show that Cronbach's alpha value is 0.784, which is within a reasonable reliability interval, indicating that the content and evaluation reliability of the “Classroom Observation Record Form” in this study is good, and the results of this study can be used.

Secondly, the validity of the scale was analyzed by factor analysis. The result is as shown in Table 2.

The results of the report show that the KMO metric value is 0.768, indicating that the evaluation system of the “Classroom Observation Record Form” in this study is suitable for factor analysis, that is, the method and content of this study are more reasonable and accurate.

## 4. Results Analysis and Discussion

### 4.1. Results and Analysis

Through the observation and analysis of 100 music performance classes, the researchers presented and discussed the scores of the observation table in the classroom records. After comparing the excellent courses at the ministerial level with the daily courses, the observation table was integrated and the observation indicators were decomposed step by step and refined as follows: A more specific and intuitive observation point is to focus on various teaching links such as classes, activities, and evaluations through observation points to ensure information technology and musicology combining the landing of the subject with the teaching level provides the observer with an operable path and method as shown in Table 3.

This study uses SPSS software to conduct nonparametric test analysis on the scores of 50 excellent courses and 50 daily courses. From the test report, it can be concluded that the asymptotic significance value of “using integrated technology to present the content characteristics of teaching materials” is 0.309; the asymptotic significance value of “presenting the learning points of knowledge and skills with integrated technology” is 0.052; the asymptotic significance value of “learning evaluation with integrated technology” is 0.096. The asymptotic significance values of the three observation indicators are all greater than 0.05, so there is no significant difference between the excellent course and the daily course. The asymptotic significance values of the other four observation indicators are all less than 0.05, so there is a significant difference between the excellent course and the daily course.

After combining the observation table and data analysis results, this paper presents the content characteristics of the textbook through integrated technology, the learning points of knowledge and skills through integrated technology, the integrated technology to create learning situations, the integrated technology to solve the learning difficulties, the integrated technology to regulate the learning process, and the integrated technology carrying out learning evaluation, integrating technology to mobilize classroom participation, a total of three observation dimensions, seven observation indicators, and related application effectiveness parts are discussed and analyzed to investigate and judge the differences between ministerial-level excellent teachers and daily teachers in multimedia teaching applications.

### 4.2. Analysis of the Characteristics of Multimedia Teaching Design

In this section, the results of each observation index under the three dimensions of the multimedia teaching application design for music performance teachers are counted and summarized, and the results are analyzed by synthesizing the relevant indicators of each dimension.

From Table 4, it can be concluded that the number of excellent, good, qualified, and required effort scores of the teachers of the Ministry of Education is 26, 21, 3, and 0, respectively, accounting for 52%, 42%, 6%, and 0% of the total sample; The number of teachers' scores in excellent, good, qualified, and effort required is 23, 19, 6, and 2, respectively, accounting for 46%, 38%, 12%, and 4% of the sample. The score intervals of the two are mainly distributed in two aspects: 4 points and 3 points. The results are in line with the assumptions of the SPSS nonparametric test analysis. There is little difference in the content characteristics of the teaching materials presented by the excellent teachers and the daily teachers. Most are doing well.

The research data shows that the teachers of both types of courses focus on the premise of effectively carrying out classroom teaching, analyze the teaching content, and present the characteristics of the content and knowledge of the teaching materials. Most of the multimedia applications of ministerial-level excellent courses are based on an intuitive image, grasp the content learning level, and allow college students to perceive the specific content of specific music phenomena. In the process of music learning in the same course, the teachers of daily lessons also use multimedia teaching design, and can also display the specific content knowledge intuitively and accurately. Students can quickly understand the purpose of the teacher's teaching content, and effectively listen and appreciate learning to achieve the emotion of music. It is understood that in the end, the students' responses in this part of the learning experience are relatively ideal.

Therefore, in presenting the content of the teaching materials, the multimedia design should clearly and accurately grasp the characteristics of the teaching materials, so that the students can concentrate on their thinking, naturally guide the students to appreciate and understand music, explore the culture of audio music, and follow the teacher's design content to initially understand the basic rhythm, speed, emotion, etc. of the teaching materials. The inner human emotion is contained in style and music.

### 4.3. Comparative Analysis of Multimedia Classroom Teaching Application Behavior

By presenting the data and arranging the data, the author finds that there are commonalities and differences in the application of multimedia teaching by excellent teachers and daily teachers in the context of integrating the subject knowledge of information technology.

From Figure 3, it can be concluded that the average scores of the seven observation indicators of the excellent teachers in the department are higher than those of the teachers in the daily lessons. Among them, the two are “using integrated technology to present the content characteristics of textbooks” and “using integrated technology to present knowledge-capable learning.” The performances of three aspects of “Key Points” and “Using Integrated Technology to Carry out Learning Evaluation” are relatively close. The performance of four aspects of integrating technology to mobilize classroom participation is quite different. The results were consistent with the assumptions of the SPSS nonparametric test analysis. The research shows that the teachers with excellent courses can reflect the characteristics of multimedia teaching applications serving the classroom, and the teaching application effect is good. In terms of “presenting the content of teaching materials,” teachers in daily classes can also carry out the teaching process around the teaching content, but the overall effect of multimedia teaching application is lower than that of teachers of excellent courses. From the overall observation of the effectiveness of music performance teachers' multimedia teaching application in one hundred classroom records, it can reflect the common points of music teachers' multimedia application teaching experience and the significant differences in teachers' multimedia application.

### 4.4. Improving the Understanding and Deepening of Music Performance Skills

Judging from the overall average scores of the two class tests, the average score of the class that implements technology-integrated learning is 7 points higher than the average score of the class that implements receptive learning. The understanding of conceptual knowledge can play a more positive role. Second, judging from the distribution of the number of students in each grade, in the classes that implement technology-integrated learning, the number of students in the high-score segment is significantly larger than that in the receptive learning class (in “81–90” and “91”∼100” is 4 and 3 people higher in these two fractions). It can be seen that for most students, information technology-integrated learning can mobilize their enthusiasm for learning and improve the effect and quality of learning. In addition, during the author's later interviews, we also found that a considerable number of students believe that information technology-integrated learning is helpful for them to comprehend some abstract concepts and theoretical knowledge. Mutual communication, discussion, and sharing through QQ groups, virtual learning communities, and other forms play an important role in eliminating doubts in the minds of different learners. Specific knowledge also deepens the learner's understanding and mastery of knowledge as shown in Figure 4.

Judging from students' performance in classroom performance, the class that implements technology-integrated learning is more engaged, has a better standard, and delicate than the class that implements receptive learning. This is not only reflected in the students' grasp of different musical instrument performance skills, but it is also reflected in the students' understanding of different musical emotions, as well as the team's tacit understanding and cooperation in cooperative performance, as shown in Figure 5.

In terms of the complete quality of students' work, the class that implements technology-integrated learning has higher completion quality than the class that implements receptive learning, especially on the evaluation scale of “excellent,” the former is 23 points higher than the latter with 3 percentage points higher on the “good” rating scale. On the whole, the students in the technology-integrated learning class are more proficient in live performance skills and later music processing skills than the students in the receptive learning class. Judging from the completion of the works, most of the excellent, complete, and innovative performance works are from classes that implement technology-integrated learning. In addition, the students themselves reported that technology-integrated learning gave them more opportunities for practical operation and simulation training, and more channels to solve their doubts. Virtual learning communities, Baidu search, related discussion QQ groups, WeChat groups, etc., are highly used forms of communication and learning.

## 5. Conclusion

The application of multimedia in music performance teaching is very extensive. It is an important teaching form under the current curriculum reform and diversified teaching trend. Teachers can convey music performance education information to students in an all-around way through multimedia teaching. It is very important for students to accept knowledge happily in the process of learning. Through the study of music knowledge, students' music literacy can be improved and their music appreciation ability can be exercised.

The application of this research is not to compare the pros and cons of the multimedia teaching of the excellent teachers and the daily teachers, but to observe and analyze the multimedia teaching process of the music performance classroom through the classroom observation perspective of TPACK. It can better improve the classroom teaching efficiency of music performance teachers. Based on the data comparison, the author summarizes and sorts out the main research results and reflects suggestions on the application of multimedia teaching for music performance teachers.

Teachers must first have a deep understanding and excavation of the teaching theme and understand how to select the appropriate type or form of multimedia teaching technology as support, in order to correctly use multimedia teaching according to different teaching contents. Teachers should learn to judge what kind of multimedia should be used in actual teaching and how to use it effectively, including the design of classroom content, layout, and format, and choose the most suitable multimedia teaching method according to different teaching topics.

Teachers' multimedia teaching experience originates from classroom practice and is continuously improved and developed in teaching practice. The integration of multimedia teaching application and teaching activity practice from the perspective of TPACK needs to run through every teaching process in teaching presupposition, teaching implementation, teaching reflection, and teaching evaluation. Only in this way can teachers promote the progress and perfection of multimedia teaching applications under the subject teaching knowledge of integrated technology.

## Figures and Tables

**Figure 1:** Schematic diagram of research architecture.

**Figure 2:** TPACK theoretical framework.

**Figure 3:** Statistics chart of the average score of observation indicators of excellent courses and daily courses.

**Figure 4:** The distribution of the number of people with different scores in the thematic test of musical performance theory knowledge.

**Figure 5:** Distribution of evaluation grades for completed works.

**Table 1:** List of feasibility statistics reports for the average scores of excellent courses and daily courses.

Cronbach's alpha	Items
0.784	7

**Table 2:** List of KMO and Bartlett test reports.

Kaiser–Meyer–Olkin-metric of sampling adequacy		0.768
Sphericity test of Bartlett	Approximate chi-square	214.34
	df	21
	Sig	0.000

**Table 3:** SPSS analysis report for the observation index scores of excellent courses and daily courses.

Category	Use integrated technology to present the content characteristics of teaching materials	Learning points for presenting knowledge skills with integrated technology	Creating learning situations with integrated technology	Solve learning difficulties with integrated technology	Regulating the learning process with integrated technology	Learning assessment using integrated technology	Mobilizing classroom engagement with integrated technology
Mann–Whitney U test	1116.5	992.5	539	411.5	376.5	1026	431.5
Wilcoxon W	2391.5	2267.5	1814	1686.5	1651.5	2301	1706.5
Z	−1.018	−1.943	−5.141	−6.041	−6.396	−1.667	−5.928
Asymptotic significance (two-sided)	0.309	0.052	0.000	0.000	0.000	0.096	0.000

**Table 4:** The score statistics of “presenting the content characteristics of textbooks with integrated technology.”

	Ministry excellent course		Daily class	
	Quantity	The proportion (%)	Quantity	The proportion (%)
Excellent (4 points)	26	52	23	46
Good (3 points)	21	42	19	38
Qualified (2 points)	3	6	6	12
Must work hard (1 point)	0	0	2	4

## Data Availability

The labeled data set used to support the findings of this study is available from the corresponding author upon request.
